# Association between the Use of Biomass as Fuel for Cooking and Acute Respiratory Infections in Children under 5 Years of Age in Peru: An Analysis of a Population-Based Survey, 2019

**DOI:** 10.1155/2022/4334794

**Published:** 2022-05-20

**Authors:** Renato Chávez-Zacarías, Félix Lindo-Cavero, Brenda Caira-Chuquineyra, Daniel Fernandez-Guzman, Carolina J. Delgado-Flores, Carlos J. Toro-Huamanchumo, Diego Urrunaga-Pastor, Guido Bendezu-Quispe

**Affiliations:** ^1^Universidad Científica del Sur, Facultad de Ciencias de la Salud, Carrera de Medicina Humana, Lima, Peru; ^2^Grupo Peruano de Investigación Epidemiológica, Unidad para la Generación y Síntesis de Evidencias en Salud, Universidad San Ignacio de Loyola, Lima, Peru; ^3^Facultad de Medicina, Universidad Nacional de San Agustín, Arequipa, Peru; ^4^Escuela Profesional de Medicina Humana, Universidad Nacional de San Antonio Abad del Cusco, Cusco, Peru; ^5^Instituto de Evaluación de Tecnologías en Salud e Investigación—IETSI, EsSalud, Lima, Peru; ^6^Unidad para la Generación y Síntesis de Evidencias en Salud, Universidad San Ignacio de Loyola, Lima, Peru; ^7^Clínica Avendaño, Unidad de Investigación Multidisciplinaria, Lima, Peru; ^8^Universidad Privada Norbert Wiener, Centro de Investigación Epidemiológica en Salud Global, Lima, Peru

## Abstract

**Background:**

Acute respiratory infections (ARIs) are the most frequent respiratory diseases associated with the use of biomass as fuel within the home. ARIs are the main cause of mortality in children under 5 years of age. We aimed to evaluate the association between the use of biomass as cooking fuel and ARI in children under 5 years of age in Peru in 2019.

**Methods:**

A secondary data analysis of the 2019 Peru Demographic and Family Health Survey (ENDES) has been performed. The outcome variable was a history of ARI. The exposure variable was the use of biomass as fuel for cooking food. To evaluate the association of interest, generalized linear models from the Poisson family with logarithmic link function considering complex sampling to estimate crude prevalence ratio (cPR) and adjusted prevalence ratio (aPR) with their respective 95% confidence intervals have been performed. *P* values <0.05 were considered statistically significant.

**Results:**

A total of 16,043 children were included in the analysis. Of the total, biomass was used as fuel to cook food in the homes of 3,479 (20.0%) children. Likewise, 2,185 (14.3%) of the children had a history of ARI. In the adjusted model, it was found that children living in homes in which biomass was used as cooking fuel had a greater probability of presenting ARI (aPR = 1.13; 95% CI: 1.01–1.28).

**Conclusions:**

It has been found that biomass was used to cook food in two of every 10 households. Likewise, almost one-seventh of children under 5 years old presented an ARI. The use of biomass as a source of energy for cooking in the home was associated with a higher probability of presenting ARIs.

## 1. Introduction

Cooking food and boiling water are fundamental processes for disease prevention [1, 2]. In urban cities, one of the main sources of energy to carry out this process is the use of clean fuels (liquefied petroleum gas (LPG), electricity, biogas, ethanol gel, vegetable oils) [3, 4]. However, in rural or lower-income populations, where households cannot afford these clean fuels, a higher proportion of use of biomass fuels or pollutants such as wood, charcoal, animal manure, and agricultural residues is reported [5, 6].

In 2015, more than 3 billion people around the world relied on polluting energy sources in their homes to cook, heat their food, and light their homes [7]. The combustion of these biomass products leads to increased smoke formation, with the emission of environmental pollutants such as carbon monoxide (CO) and inhalable particulate matter (PM 10 and PM 2.5) [8]. Consequently, daily exposure to the smoke of these fuels by members of a household may represent a greater risk of mortality [9] and the appearance of acute and chronic respiratory diseases [10].

Among respiratory diseases, acute respiratory infections (ARIs) are the most frequently associated infections with the use of biomass as fuel within the home [11]. ARIs are the main cause of mortality in children under 5 years of age [12], with a global rate of 35.4% in 2017 [13]. The risk factors related to morbidity and mortality by ARI in children under 5 years of age described include being younger, being male, having a low birth weight, and low parental educational level [14, 15]. In contrast, greater vaccination coverage and reductions in household air pollution are factors that have shown a greater reduction in mortality from ARI in children under 5 years of age [16].

Taking the aforementioned into account, the purpose of this study was to evaluate the association between the use of biomass as cooking fuel and the prevalence of ARIs in children under 5 years of age in Peru in 2019. This study aimed to reinforce the collective evidence on the risk of biomass use in households and promote the formulation of measures that could reduce exposure to biomass fuel among local and national political decision-makers.

## 2. Material and Methods

### 2.1. Study Design

A secondary analysis of data from the 2019 Peru Demographic and Family Health Survey (ENDES) has been carried out, which is developed annually through the National Institute of Statistics and Informatics (INEI). The ENDES includes three questionnaires: the household questionnaire, the individual woman questionnaire, and the health questionnaire. The household questionnaire was used for this study.

### 2.2. Population, Sample, and Sampling

This survey is representative at the urban-rural, regional, and national levels. The ENDES is a multistage survey with a probabilistic sampling design by conglomerates and stratified at the departmental level and by urban and rural areas. The primary sampling unit is made up of selected clusters. The secondary sampling unit was the selected dwellings. Additional information on the ENDES survey methodology is available in the technical report [17].

A total of 20,937 mothers of children between 0 and 5 years of age were surveyed with the household questionnaire in 2019. This questionnaire contains a section of questions on health characteristics of household members and basic characteristics of the home. In this study, for the analysis we only considered the mothers of children under 5 years of age who answered the questions that make up the variables of interest (ARI and use of biomass as fuel) and who had complete data on the rest of the covariates evaluated. The effective sample for our study consisted of 16,043 children under 5 years of age (Figure 1).

### 2.3. Variables

The dependent variable of the study was a history of ARI. This variable was defined as the presence of cough in the last 2 weeks and the presence of respiratory distress or short breaths. The questions “Has the child suffered from a cough in the last 2 weeks?” and “Did the child have rapid/short breaths and/or had respiratory distress in the last few weeks?” were used, for which the response options were as follows: yes, no, and don't know. A history of ARI was defined as a positive response to both questions.

The independent variable of the study was the use of biomass as fuel, which was evaluated with the following question “What is the fuel that you most frequently use in your home for cooking?” To define the variable, it was categorized into two groups: no biomass (electricity, liquid oil, natural gas, biogas, and kerosene) and biomass (charcoal, mineral charcoal, firewood, dung, agricultural residues, and reeds or shrubs).

The following covariates of interest were considered according to the previous literature [3, 18–21]: characteristics of the child: age of the child (less than 1 year, 1 year, 2 years, 3 years, and 4 years), sex of the child (male and female), size at birth (adequate, low weight, and macrosomic), lactation status (yes and no), parity (first child, second child, and third child or more), type of gestation (single and multiple), interpregnancy interval (adequate, short, and long), place of delivery (institutional and noninstitutional), type of delivery (vaginal and cesarean section), and number of prenatal check-ups (greater than or equal to six and less than six); characteristics of the home: drinking water at home (yes and no) and number of rooms (one and more than one); and mother's characteristics: mother's age (in tertiles: 12 to 26 years, 27 to 33 years, and 34 to 49 years), marital status (married or cohabiting and not married or cohabiting), level of education (primary or preschool, secondary, and higher), currently working (yes and no), health insurance (yes and no), geographic region (Metropolitan Lima, rest of the coast, highlands, and jungle), area of residence (urban and rural), level of wealth (low income (defined as the fourth and fifth wealth quintiles), middle income (defined as the third wealth quintile), high income (defined as the first and second wealth quintiles)), ethnicity (mestizo, Quechua, black or moreno or zambo, and others (Aymara, indigenous, or native of the Amazon and white)), current smoker (yes and no), intimate partner violence (yes and no), and level of education of the partner (primary or preschool, secondary, and higher).

### 2.4. Statistical Analysis

The 2019 ENDES databases were downloaded and imported into the Stata® v.16.0 program (Stata Corporation, College Station, Texas, USA) to perform the joining of bases according to the methodology described by Hernández-Vásquez et al. at [22]. All analyses were carried out considering the characteristics of the complex survey design and the weighting factors of the ENDES using the Stata “SVY” module.

For descriptive analysis, since all variables were categorical, absolute frequencies and weighted proportions were calculated. For the bivariate analysis, a comparison of the covariates was made with the history of biomass use as fuel and the history of acute respiratory infection. For this, the chi-square test with the Rao–Scott correction was used.

To evaluate the association of interest, generalized linear models of the Poisson family with logarithmic link function were used, and crude prevalence ratio (cPR) and adjusted prevalence ratio (aPR) have been calculated. For the adjusted model, the method of forward manual selection and the Wald test were used to select the variables that allow obtaining a final parsimonious model. In this way, the variables such as age, level of wealth, region, intimate partner violence, type of childbirth, and sex of the child were entered into the final model. The analyses were reported with their respective 95% confidence intervals (95% CI), and *p* values <0.05 were considered statistically significant.

### 2.5. Ethical Aspects

The protocol of this study was evaluated and accepted by the ethics committee of the *Universidad Científica del Sur* (198-2020-PRE15). The database used (ENDES) is in the public domain (http://iinei.inei.gob.pe/microdatos/). Since this database does not include data that allow the identification of the subjects surveyed, the confidentiality of the participants was ensured. The collection of primary data from this survey, carried out by the INEI team, previously required the consent of the respondents to participate [17].

## 3. Results

### 3.1. Prevalence of the Use of Biomass as Fuel for Cooking According to the Child Characteristics

A total of 16,043 children were included in the analysis (Figure 1). Most were 4 years old (21.8%), 50.5% were male, 84.0% were born with an adequate size at birth, 35.6% were the third child or more, and 91.8% and 34.0% were born by institutional delivery and cesarean section, respectively. Regarding the characteristics of the home, access to drinking water in the home was not present in 9.1% and 20.3% of children lived in places that had only one room. The prevalence of biomass used as fuel was 20.0%, while the most frequent non-biomass fuel used was LPG (90.5%), natural gas (9.1%), and electric kitchen (0.5%). Children of 3 years of age (*p*=0.030), who lived in a home without drinking water (*p* < 0.001),who had a history of being macrosomic at birth (*p* < 0.001), being the third child or more (*p* < 0.001), the product of a multiple gestation (*p* < 0.001), with short interpregnancy interval (*p* < 0.001), noninstitutional place of delivery (*p* < 0.001), born by vaginal delivery (*p* < 0.001), and with <6 prenatal visits (*p*=0.002) had a significantly higher exposure to biomass (Table 1).

### 3.2. Prevalence of the Use of Biomass as Fuel for Cooking According to the Mother Characteristics

Regarding the characteristics of the children's mothers, the majority were between 27 and 33 years old (40.1%), were married or had a partner (90.6%), 44.6% had a secondary education level, 27.3% lived in a rural area, and 52.7% reported having experienced intimate partner violence. The use of biomass as fuel for cooking was significantly more frequent in mothers aged 12 to 26 years (*p*=0.042), married or living together (*p* < 0.001), with a degree of primary or preschool education (*p* < 0.001), without work at the time of the survey (*p* < 0.001), with health insurance (*p* < 0.001), from highlands (*p* < 0.001) and rural areas (*p* < 0.001), with low income (*p* < 0.001), from an ethnic group other than mestizo, Quechua, or black/brown/zambo, were not current smokers (*p* < 0.001), and with a partner with a primary or preschool education level (*p* < 0.001) (Table 2).

### 3.3. Prevalence of a History of Acute Respiratory Infection in Children in the Last Two Weeks According to the Child Characteristics

The prevalence of ARIs in the last two weeks in children under 5 years was 14.3%. Children of 1 year of age (*p*=0.001), who were male (*p*=0.021), with an active lactation status (*p*=0.035), with short interpregnancy interval (*p*=0.012), born by cesarean section (*p*=0.017), with <6 prenatal visits (*p* < 0.001), only one room in their homes (*p*=0.010), and exposed to biomass as a fuel type used for cooking (*p*=0.030) had a significantly higher ARI prevalence (Table 3).

### 3.4. Prevalence of a History of Acute Respiratory Infection in Children in the Last Two Weeks According to the Mother Characteristics

The prevalence of ARI was more frequent in mothers aged 12 to 26 years (*p* < 0.001), not married or cohabitating (*p*=0.007), living in the jungle (*p* < 0.001), with low income (*p*=0.003), current smoker (*p*=0.012), who experienced intimate partner violence (*p* < 0.001), and with a degree of primary or preschool education (*p*=0.024) (Table 4).

### 3.5. Association between the Type of Fuel Used for Cooking and a History of Acute Respiratory Infection in Children in the Last Two Weeks

Regarding the result of the regression models, the crude model found that children living in households with biomass as fuel had a greater probability of presenting ARI compared with children in households in which biomass is not used (cPR = 1.13; 95% CI: 1.01–1.26). This association remained present in the adjusted model (aPR = 1.13; 95% CI: 1.01–1.28) (Table 5).

## 4. Discussion

### 4.1. Main Results

This study aimed to estimate the association between the use of biomass as fuel in the home and the presence of ARIs in Peruvian children under five years of age. It was found that approximately one in seven children under the age of 5 had a history of ARI in the past 14 days. The use of biomass as fuel in the home was associated with a higher probability of presenting ARI. These findings provide evidence on the influence of household air pollution on respiratory illnesses in children under five years of age.

### 4.2. Prevalence of Use of Biomass as Fuel in the Home

In Peru, 2 of every 10 children under 5 years of age are exposed to the use of biomass as fuel for cooking at home (charcoal, mineral coal, firewood, manure, agricultural residues, reeds/shrubs). It has been estimated that at a global level the energy produced by biomass represents around 14% of primary energy, being 35% in developing countries [23]. In 2017, the use of biomass worldwide was higher compared with the rest of renewable energies compared with previous years, especially in countries in Asia, Africa, and America [24]. In developing countries, it has been estimated that approximately 50% of people use biomass fuels for domestic energy [25]. It was found that in Peruvian rural areas, biomass use occurs in 60.2%. This percentage is higher than that reported in rural areas of India (50%), China (33%), and Brazil (25%) [26]. The high proportions of biomass use in rural areas are possibly due to the lower purchasing power and access to and distribution of cleaner fuels in these areas compared with urban areas.

In Peru, a reduction in the use of biomass within the home has been reported, decreasing from about 10 million inhabitants in 2010 [27] to almost 6 million in 2017 [28]. This decrease in biomass use could be due to the creation of laws and programs to guarantee universal access to clean fuel (LPG) through the implementation of modern kitchens since 2012, which would guarantee less pollution production inside homes [29, 30]. Chronic exposure to high levels of PM 2.5 and PM 10, products generated from biomass burning, is related to higher morbidity and mortality by various causes [31–33]. Therefore, it is necessary to increase the purchase and distribution of cleaner fuels in the homes of the country, ensuring a reasonable price for the most vulnerable populations, such as those located in rural areas.

### 4.3. Prevalence of ARIs

It has been found that in 2019 nearly one in seven children under 5 years had ARIs. A systematic review of studies conducted in Ethiopia reported a prevalence of 17.3%, the predictors of which were holding the child on the back during food preparation and the use of non-energy sources for cooking [34]. Likewise, a global analysis reported that the prevalence of respiratory symptoms ranged between 3.4% and 7.9% in Africa and 12.5% in Latin America and the Caribbean [35]. The risk predictors in this study were a high level of PM 2.5 environmental contamination, low socioeconomic status, the presence of smokers in the home, and low birth weight [35]. This is similar to what was found in our study, in which the highest proportion of ARIs was found among children aged one year or less than one-year-old, of unmarried or cohabiting mothers, who smoke, and with a low educational or economic level. Therefore, the need to reduce ARIs and their associated consequences should be reinforced through the promotion of breastfeeding, full coverage for immuno-preventable diseases, and epidemiological surveillance, among other proposals, because these are measures that have been shown to reduce the ARI rates [36].

### 4.4. Use of Biomass as Fuel and IRAs

A higher prevalence of ARIs in children under 5 years of age in households that used compared with those that did not use biomass as fuel has been found. After adjusting for confounders in the multivariate model, a significant association was found between these variables, which is consistent with previous studies [11, 37]. In this age group (under 5 years of age), which has greater immunological susceptibility to infection, a greater risk of hospital admissions due to ARIs has been reported compared with other age groups also exposed to biomass burning [38].

Biomass burning inside homes generates high-magnitude concentrations of harmful substances such as CO (an 8-hour average: about 40.7 ppm SD: 40.0 ppm), PM 2.5, and PM 10, exceeding World Health Organization (WHO) Indoor Air Quality Standards [39, 40]. This stimulates an inflammatory response in the airways [41, 42] and greater tissue damage favoring the development of respiratory diseases [32]. This would explain the effects that domestic air pollution has on health, which is why it is a problem for global public health and requires greater efforts in the areas of prevention and mitigation through the formulation of policies, with special emphasis on rural zones.

### 4.5. Implications for Public Health

ARIs are the main cause of morbidity and mortality among children under 5 years of age [12, 36]. The findings of this study suggest a potential impact of domestic air pollution on the prevalence of ARIs in this population. In Peru, the effect of the use of biomass as fuel in the home has a strong impact on public health, since it is related to a series of medical conditions such as respiratory diseases, neonatal morbidity and mortality, heart disease, and neoplasms [43, 44], and this study has been associated with greater development of ARIs.

The positive effect of using alternative clean energy sources and the improvement of stoves and behavioral interventions on maternal and child health has been previously described in the literature [45–47], decreasing the proportion of acute respiratory diseases in children under 5 years of age.

In Peru, about 1,800,000 families and 70.8% of the rural population still use biomass to cook their food [43]. In this regard, Law 29852, created in 2012, established the Social Energy Inclusion Fund (FISE) [29] with the objective of providing the infrastructure required for the security of the energy system and ensuring universal access to energy. Likewise, this law sought to promote access to LPG through the creation of the “Programa de compensación social y promoción para el acceso al GLP” [30], and to implement modern cooking in homes, so that by 2030 all Peruvian households can cook with clean fuels according to the Sustainable Development Goals [48].

ARIs can be prevented through interventions that allow good coverage of immunizations, diet, and control of environmental factors [36]. In Peru, a health directive has been established for the epidemiological surveillance of ARIs that is applied on a mandatory basis in all health facilities nationwide [49]. For this reason, it is important to manage environmental factors, such as the use of biomass as fuel, which could increase the prevalence of respiratory diseases.

### 4.6. Strengths and Limitations

Although our results are compatible with what was reported in previous studies [3, 5, 11, 19], the following limitations should be considered in this study. First, it must be recognized that, despite having found in our study an association between the use of biomass as fuel in the home and a history of ARIs, causality cannot be established because temporality is lacking due to the cross-sectional design of the survey. However, our outcome variable evaluated the presence of ARIs in the last 14 days, and it is unlikely that the use of biomass as cooking fuels has varied considerably in this period of time. Second, when the data evaluated come from a secondary database, other factors related to the child (such as children's exposure time and proximity to the stove or kitchen during food cooking), aspects of the home (such as the location of the kitchen and kitchen ventilation), and factors related to the environment (such as environmental pollution where the dwellings are located) of interest were not included in the measurements carried out by ENDES. Third, there may have been recall bias or social desirability bias in the questionnaire questions collected by self-reporting. Despite these limitations, the ENDES is a survey of national and regional representativeness, which is carried out annually following methodological quality control processes, and the use of the database of this survey allows for evaluating health information of children under 5 years of age and the characteristics of the household. Likewise, previous studies in other countries have used demographic and health surveys similar to the ENDES to study the use of biomass and ARIs [3, 18–21], and thus, this type of survey is a useful data source for the subject studied. Therefore, consider that the findings of this study can provide an overview of the association between domestic air pollution and ARI in Peruvian children under 5 years of age.

## 5. Conclusion

In Peru, 1 in 7 children under the age of 5 presented ARIs in the last 14 days, with the use of biomass as fuel in the home being associated with a higher prevalence of ARIs. Therefore, the need to implement strategies or support programs that ensure access to clean fuel in the home is reinforced, prioritizing rural and indigenous populations to reduce the prevalence of acute respiratory diseases in children under 5 years of age.

## Figures and Tables

**Figure 1:** Flow chart for sample selection.

**Table 1:** Prevalence of the use of biomass as fuel for cooking according to the child characteristics (*n* = 16,043).

Characteristics	Total		Type of fuel used in cooking				*Pvalue*
			Biomass		No biomass		
	n (%^*∗*^)	95% CI^*∗*^	n (%^*∗*^)	95% CI^*∗*^	n (%^*∗*^)	95% CI^*∗*^	
	16,043 (100)		3,479 (20.0)		12,564 (80.0)		
Child characteristics							
Age							0.030
Under 1 year	2,750 (16.7)	16.0–17.4	615 (21.1)	19.3–23.1	2,135 (78.9)	76.9–80.7	
1 year	3,171 (19.9)	19.2–20.7	676 (19.3)	17.6–21.0	2,495 (80.7)	79.0–82.4	
2 years	3,251 (20.3)	19.5–21.1	643 (18.1)	16.5–19.8	2,608 (81.9)	80.2–83.5	
3 years	3,398 (21.3)	20.5–22.1	793 (21.2)	78.1–81.4	2,605 (78.8)	77.0–80.5	
4 years	3,473 (21.8)	21.1–22.6	752 (20.2)	18.6–21.8	2,721 (79.8)	78.2–81.4	
Sex							0.139
Male	8,219 (50.5)	49.6–51.5	1,742 (19.4)	18.3–20.6	6,477 (80.6)	79.4–81.7	
Female	7,824 (49.5)	48.5–50.4	1,737 (20.5)	19.3–21.7	6,087 (79.5)	78.3–80.7	
Size at birth							<0.001
Adequate	13,500 (84.0)	83.1–84.8	2,747 (18.3)	17.3–19.3	10,753 (81.7)	80.7–82.7	
Underweight	940 (5.8)	5.3–6.3	271 (28.2)	24.3–32.3	669 (71.9)	67.7–75.7	
Macrosomic	1,603 (10.2)	9.5–10.9	461 (29.2)	25.6–33.0	1,141 (70.8)	67.0–74.4	
Lactation status							0.900
No	10,381 (64.6)	63.7–65.5	2,219 (20.0)	18.9–21.1	8,162 (80.0)	78.9–81.1	
Yes	5,662 (35.4)	34.5–36.3	1,260 (19.9)	18.6–21.3	4,402 (80.1)	78.7–81.4	
Parity							<0.001
First child	4,863 (31.2)	30.3–32.1	729 (13.8)	12.6–15.0	4,134 (86.3)	85.0–87.4	
Second child	5,313 (33.2)	32.4–34.1	818 (14.1)	13.0–15.2	4,495 (85.9)	84.8–87.0	
Third child or more	5,867 (35.6)	34.6–36.6	1,932 (30.9)	29.1–32.7	3,935 (69.1)	67.3–70.9	
Type of pregnancy							<0.001
Only	15,774 (98.5)	98.1–98.8	3,396 (19.7)	18.7–20.7	12,378 (80.3)	79.3–81.3	
Multiple	2,69 (1.5)	1.2–1.9	83 (37.1)	27.3–48.2	186 (62.9)	51.8–72.7	
Interpregnancy interval							<0.001
Adequate	5,079 (31.8)	30.9–32.7	1,386 (25.5)	23.7–27.4	3,693 (74.5)	72.6–76.3	
Short	410 (2.6)	2.3–2.9	123 (30.1)	24.9–25.8	287 (69.9)	64.2–75.1	
Long	10,554 (65.6)	64.6–66.6	1,970 (16.9)	16.0–17.8	8,584 (83.1)	82.2–84.0	
Place of delivery							<0.001
Institutional	14,904 (91.8)	90.9–92.5	2,761 (16.2)	15.3–17.1	12,143 (83.8)	82.9–84.7	
Noninstitutional	1,139 (8.2)	7.5–9.1	718 (62.1)	57.5–66.5	421 (37.9)	33.5–42.5	
Delivery type							<0.001
Vaginal	10,856 (66.0)	64.9–67.1	2,949 (25.7)	24.4–27.1	7,907 (74.3)	72.9–75.6	
Cesarean	5,187 (34.0)	32.9–35.1	530 (8.8)	7.7–9.9	4,657 (91.2)	90.1–92.3	
Number of prenatal visits							0.002
≥6	14,911 (92.9)	92.4–93.4	3,186 (19.6)	18.7–20.6	11,725 (80.4)	79.4–81.3	
<6	1,132 (7.1)	6.6–7.6	293 (24.1)	21.1–27.4	839 (75.9)	72.6–78.9	
Home characteristics							
Drinking water at home							<0.001
Yes	14,751 (90.9)	89.7–92.0	2,834 (17.3)	16.3–18.3	11917 (82.7)	81.7–83.7	
No	1,292 (9.1)	8.0–10.3	645 (46.7)	40.9–52.5	647 (53.3)	47.5–59.1	
Number of rooms							0.363
One	3,491 (20.3)	19.4–21.2	768 (20.8)	18.8–22.8	2,723 (79.3)	77.2–81.2	
More than one	12,552 (79.7)	78.8–80.6	2,711 (19.7)	18.7–20.9	9,841 (80.3)	79.1–81.3	

^*∗*^Percentages weighted according to the complex sampling design.

**Table 2:** Prevalence of the use of biomass as fuel for cooking according to the characteristics of the mother (*n* = 16,043).

Characteristics	Total		Type of fuel used in cooking				*Pvalue*
			Biomass		No biomass		
	n (%^*∗*^)	95% CI^*∗*^	n (%^*∗*^)	95% CI^*∗*^	n (%^*∗*^)	95% CI^*∗*^	
	16,043 (100)		3,479 (20.0)		12,564 (80.0)		
Age							0.042
12–26 years	4,935 (30.2)	29.2–31.3	1,069 (21.2)	19.5–23.0	3,866 (78.8)	77.0–80.5	
27–33 years	6,490 (40.1)	39.1–41.2	1,324 (18.7)	17.4–20.0	5,166 (81.3)	79.9–82.6	
34–49 years	4,618 (29.7)	28.7–30.7	1,086 (20.4)	18.8–22.0	3,532 (79.6)	78.0–81.2	
Marital status							<0.001
Married/cohabiting	14,464 (90.6)	89.9–91.2	3,218 (20.5)	19.5–21.6	11,246 (79.5)	78.4–80.5	
Not married/cohabiting	1,579 (9.4)	88.3–10.1	261 (14.7)	12.6–17.1	1,318 (85.3)	82.9–87.4	
Degree of instruction							<0.001
Primary or preschool	3,253 (20.4)	19.4–21.3	1,790 (53.9)	51.2–56.7	1,463 (46.1)	43.3–48.8	
Secondary	7,323 (44.6)	43.4–45.7	1,459 (17.6)	16.3–18.9	5,864 (82.4)	81.1–83.7	
Higher	5,467 (35.0)	33.9–36.2	230 (3.2)	2.5–4.1	5,237 (96.8)	95.9–97.5	
Currently works							<0.001
Yes	10,614 (65.1)	63.9–66.3	2,253 (18.6)	17.5–19.8	8,361 (81.4)	80.2–82.5	
No	5,429 (34.9)	33.7–36.1	1,226 (22.5)	20.8–24.3	4,203 (77.5)	75.7–79.2	
Health insurance							<0.001
Yes	13,381 (82.1)	81.2–83.0	3,237 (22.5)	21.3–23.6	10,144 (77.5)	76.4–78.7	
No	2,662 (17.9)	17.0–18.8	242 (8.5)	7.0–10.1	2,420 (91.6)	89.9–93.0	
Region							<0.001
Metropolitan Lima	1,939 (27.0)	25.9–28.1	1 (0.1)	0.0–0.3	1,938 (99.9)	99.6–99.9	
Rest of the coast	4,789 (26.3)	25.1–27.4	261 (9.1)	7.4–11.0	4,528 (91.0)	89.0–92.6	
Highlands	5,307 (28.7)	27.4–30.1	2,071 (39.3)	36.9–41.7	3,236 (60.7)	58.3–63.1	
Jungle	4,008 (18.0)	17.0–19.1	1,146 (34.8)	31.8–37.8	2,862 (65.3)	62.2–68.2	
Home							<0.001
Urban	11,439 (72.7)	71.7–73.6	684 (4.8)	4.3–5.4	10,755 (95.2)	94.6–95.7	
Rural	4,604 (27.3)	26.4–28.3	2,795 (60.2)	57.2–63.0	1,809 (39.8)	37.0–42.8	
Wealth level							<0.001
Low income	8,706 (49.7)	48.5–50.9	3,435 (39.7)	37.9–41.5	5,271 (60.3)	58.5–62.1	
Medium income	3,266 (20.0)	19.1–21.0	40 (1.1)	0.7–1.7	3,226 (98.9)	98.3–99.3	
High income	4,071 (30.3)	29.1–31.5	4 (0.0)	0.0–0.1	4,067 (99.9)	99.9–100.0	
Ethnicity							<0.001
Mestizo	6,684 (44.9)	43.7–46.1	708 (10.5)	9.4–11.7	5,976 (89.5)	88.3–90.6	
Quechua	4,593 (24.5)	23.5–25.5	1,459 (25.9)	23.9–27.9	3,134 (74.1)	72.1–76.1	
Black/moreno/zambo	1,670 (11.8)	11.0–12.6	440 (28.2)	25.1–31.5	1,230 (71.8)	68.5–74.9	
Others	3,096 (18.8)	17.8–19.9	872 (29.5)	26.7–32.6	2,224 (70.5)	67.4–73.3	
Current smoker							<0.001
No	15,788 (98.1)	97.7–98.4	3,468 (20.3)	19.3–21.3	12,320 (79.7)	78.7–80.7	
Yes	255 (1.9)	1.6–2.3	11 (2.4)	1.2–5.1	244 (97.6)	94.9–98.8	
Intimate partner violence							0.429
No	7,518 (47.1)	46.0–48.3	1,603 (20.3)	18.9–21.8	5,915 (79.7)	78.2–81.1	
Yes	8,525 (52.9)	51.7–54.0	1,876 (19.6)	18.4–20.8	6,649 (80.4)	79.2–81.6	
Degree of education of the couple							<0.001
Primary or preschool	2,376 (15.3)	14.5–16.3	1,346 (56.1)	53.0–59.1	1,030 (43.9)	40.9–47.0	
Secondary	7,848 (48.5)	47.3–50.0	1,778 (20.0)	18.7–21.3	6,070 (80.0)	78.7–81.3	
Higher	5,819 (36.2)	35.0–37.3	355 (4.6)	3.8–5.5	5,464 (95.4)	94.5–96.1	

^*∗*^Percentages weighted according to the complex sampling design.

**Table 3:** Prevalence of a history of acute respiratory infection in children in the last two weeks according to the child characteristics (*n* = 16,043).

Characteristics	Acute respiratory infection of the child in the last two weeks				*Pvalue*
	Yes		No		
	n (%^*∗*^)	95% CI^*∗*^	n (%^*∗*^)	95% CI^*∗*^	
	2,185 (14.3)		13,858 (85.7)		
Child characteristics					
Age					0.001
Under 1 year	412 (15.1)	13.4–16.9	2,338 (84.9)	83.1–86.6	
1 year	515 (16.9)	15.2–18.7	2,656 (83.1)	81.3–84.8	
2 years	395 (12.4)	11.0–13.9	2,856 (87.6)	86.1–89.0	
3 years	446 (14.2)	12.6–15.9	2,952 (85.8)	84.1–87.4	
4 years	417 (13.5)	12.0–15.1	3,056 (86.5)	84.9–88.0	
Sex					0.021
Male	1,184 (15.2)	14.1–16.3	7,035 (84.8)	83.7–85.9	
Female	1,001 (13.5)	12.6–14.5	6,823 (86.5)	85.5–87.4	
Size at birth					0.426
Adequate	1,820 (14.3)	13.5–15.1	11,680 (85.7)	84.9–86.5	
Underweight	144 (16.2)	13.4–19.4	796 (83.8)	80.6–86.6	
Macrosomic	221 (14.0)	12.0–16.3	1,382 (86.0)	83.7–88.0	
Lactation status					0.035
No	1,352 (13.8)	12.9–14.7	9,029 (86.2)	85.3–87.1	
Yes	833 (15.4)	14.2–16.6	4,829 (84.6)	83.4–85.8	
Parity					0.544
First child	681 (14.1)	12.9–15.4	4,182 (85.9)	84.5–87.1	
Second child	723 (14.9)	13.7–16.2	4,590 (85.1)	83.8–86.3	
Third child or more	781 (14.1)	12.9–15.3	5,086 (85.9)	84.7–87.1	
Type of pregnancy					0.582
Only	2,148 (14.3)	13.6–15.1	13,626 (85.7)	84.9–86.4	
Multiple	37 (16.0)	10.7–23.1	232 (84.0)	76.9–89.3	
Interpregnancy interval					0.012
Adequate	694 (15.0)	13.7–16.3	4,385 (85.1)	83.7–86.3	
Short	66 (20.3)	15.4–26.2	344 (79.7)	73.8–84.6	
Long	1,425 (13.8)	13.0–14.7	9,129 (86.2)	85.3–87.0	
Place of delivery					0.077
Institutional	2,016 (14.1)	13.4–14.9	12888 (85.9)	85.1–86.6	
Noninstitutional	169 (16.6)	14.0–19.6	970 (83.4)	80.4–86.0	
Delivery type					0.017
Vaginal	1,,438 (13.7)	12.8–14.6	9,418 (86.3)	85.4–87.2	
Cesarean section	747 (15.7)	14.3–17.1	4,440 (84.3)	82.9–85.7	
Number of prenatal visits					<0.001
≥6	1984 (14.0)	13.2–14.7	12,927 (86.0)	85.2–86.7	
<6	201 (18.8)	16.0–21.9	931 (81.2)	78.1–84.0	
Characteristics of the home					
Drinking water at home					0.239
Yes	1,976 (14.2)	13.4–15.0	12,775 (85.8)	85.0–86.6	
No	209 (15.7)	13.4–18.5	1,083 (84.3)	81.5–86.6	
Number of rooms					0.010
One	512 (16.2)	14.6–19.7	2,979 (83.8)	82.1–85.4	
More than one	1,673 (13.9)	13.1–14.7	10,879 (86.1)	85.3–86.9	
Type of fuel used for cooking					0.030
No biomasses	1,667 (14.0)	13.2–14.8	10,897 (86.0)	85.2–86.8	
Biomass	518 (15.8)	14.3–17.4	2,961 (84.2)	82.6–85.7	

^*∗*^Percentages weighted according to the complex sampling design.

**Table 4:** Prevalence of a history of acute respiratory infection in children in the last two weeks according to the characteristics of the mother (*n* = 16,043).

Characteristics	Acute respiratory infection of the child in the last two weeks				*Pvalue*
	Yes		No		
	n (% ^*∗*^)	95% CI ^*∗*^	n (% ^*∗*^)	95% CI ^*∗*^	
	2,185 (14.3)		13,858 (85.7)		
Age					<0.001
12–26 years	752 (16.0)	14.7–17.3	4,183 (84.0)	82.7–85.3	
27–33 years	887 (14.6)	13.4–15.8	5,603 (85.4)	84.2–86.6	
34–49 years	546 (12.4)	11.1–13.7	4,072 (87.6)	86.3–88.9	
Marital status					0.007
Married/cohabiting	1,938 (14.0)	13.3–14.8	12,526 (86.0)	85.2–86.7	
Not married/cohabiting	247 (17.4)	15.0–20.2	1,332 (82.6)	79.8–85.0	
Degree of instruction					0.188
Primary or preschool	482 (15.3)	13.8–16.9	2,771 (84.7)	83.1–86.2	
Secondary	1,014 (14.6)	13.6–15.7	6,309 (85.4)	84.3–86.4	
Higher	689 (13.5)	12.3–14.8	4,778 (86.5)	85.2–87.8	
Currently works					0.686
Yes	1,458 (14.4)	13.6–15.4	9,156 (85.6)	84.6–86.4	
No	727 (14.1)	13.0–15.4	4,702 (85.9)	84.6–87.0	
Health insurance					0.857
Yes	1,854 (14.4)	13.6–15.2	11,527 (85.6)	84.8–86.4	
No	331 (14.2)	12.4–16.2	2,331 (85.8)	83.8–87.6	
Region					<0.001
Metropolitan Lima	293 (15.4)	13.6–17.3	1,646 (84.6)	82.7–86.4	
Rest of the coast	566 (12.7)	11.4–14.0	4,223 (87.3)	86.0–88.6	
Highlands	677 (13.0)	11.9–14.2	4,630 (87.0)	85.8–88.1	
Jungle	649 (17.3)	15.8–19.0	3,359 (82.7)	81.0–84.2	
Home					0.077
Urban	1,513 (13.9)	13.1–14.8	9,926 (86.1)	85.2–86.9	
Rural	672 (15.4)	14.0–17.0	3,932 (84.6)	83.0–86.0	
Wealth level					0.003
Low income	1,281 (15.6)	14.7–16.7	7,425 (84.4)	83.3–85.3	
Medium income	427 (13.7)	12.2–15.4	2,839 (86.3)	84.6–87.8	
High income	477 (12.7)	11.3–14.2	3,594 (87.3)	85.8–88.7	
Ethnicity					0.485
Mestizo	912 (14.2)	13.2–15.4	5,772 (85.8)	84.6–86.8	
Quechua	620 (13.8)	12.5–15.3	3,973 (86.2)	84.8–87.5	
Black/moreno/zambo	238 (15.8)	13.7–18.3	1,432 (84.2)	81.7–86.3	
Others	415 (14.4)	12.8–16.2	2,681 (85.6)	83.8–87.2	
Current smoker					0.012
No	2,139 (14.2)	13.5–15.0	13,649 (85.8)	85.0–86.5	
Yes	46 (21.3)	15.6–28.3	209 (78.7)	71.7–84.4	
Intimate partner violence					<0.001
No	854 (11.9)	10.9–12.9	6,664 (88.1)	87.1–89.1	
Yes	1,331 (16.5)	15.5–17.6	7,194 (83.5)	82.4–84.5	
Degree of education of the couple					0.024
Primary or preschool	360 (16.1)	14.3–18.1	2,016 (83.9)	81.9–85.7	
Secondary	1,100 (14.7)	13.6–15.8	6,748 (85.3)	84.2–86.4	
Higher	725 (13.2)	12.0–14.4	5,094 (86.8)	85.6–88.0	

^*∗*^Percentages weighted according to the complex sampling design.

**Table 5:** Regression models to evaluate the association between the type of fuel used for cooking and a history of acute respiratory infection in children in the last two weeks, ENDES 2019.

Characteristics	Crude model			Adjusted epidemiological model^*∗*^		
	cPR	95% CI	*P* value	aPR	95% CI	*P* value
Type of fuel used for cooking						
No biomass	Reference			Reference		
Biomass	1.13	1.01–1.26	0.036	1.13	1.01–1.28	**0.044**

cPR: crude prevalence ratio; aPR: adjusted prevalence ratio. The prevalence ratios and confidence intervals were calculated considering the complex sampling design. *P* values < 0.05 are in bold. ^*∗*^Adjusted for age, wealth level, region, intimate partner violence, type of childbirth, and sex of the child.

## Data Availability

The database used is in the public domain (http://iinei.inei.gob.pe/microdatos/).
